# Clinical Significance, Cellular Function, and Potential Molecular Pathways of CCT7 in Endometrial Cancer

This article has been retracted.

**DOI:** 10.3389/fonc.2020.01468

**Published:** 2020-08-28

**Authors:** Liwen Wang, Wei Zhou, Hui Li, Hui Yang, Nianchun Shan

**Affiliations:** ^1^Department of Gynecology and Obstetrics, Xiangya Hospital, Central South University, Changsha, China; ^2^Xiangya School of Medicine, Central South University, Changsha, China; ^3^Department of Reproductive, Xiangya Hospital, Central South University, Changsha, China

**Keywords:** endometrial cancer, CCT7, myometrial invasion, FIGO stage, overall survival

## Abstract

**Objective:** Endometrial cancer (EC) is a common gynecologic malignancy; myometrial invasion (MI) is a typical approach of EC spreads and an important index to assess tumor metastasis and outcome in EC patients. CCT7 is a member of the TCP1 chaperone family, involved in cytoskeletal protein folding and unfolding. In this study, the role of CCT7 in EC development was investigated.

**Methods:** Clinical data for 87 EC cases and expression of CCT7 were analyzed. *CCT7* was knocked out using siRNA-*CCT7* in Ishikawa and RL95-2 cells, and their function about proliferation, apoptosis, and invasion was further tested. Bioinformatics methods were used to predict the potential pathways of *CCT7* in EC development.

**Results:** The rates of CCT7-positive cells in EC and adjacent normal endometrium tissues had a significant difference (67.8 vs. 51.4%, *p* = 0.035), and the expression rate increased from low to high pathological stage (39.7% in the I/II stage, 71.4% in the III/IV stage, *p* = 0.029). A similar change was found in protein level. CCT7 expression differed significantly between the deep MI group (>1/2) and the superficial MI group (≤1/2) (*p* = 0.039). However, there were no differences with respect to age, pathological type, and histological grade. *CCT7* suppression induced a function loss in both Ishikawa and RL95-2 cells. Bioinformatics analysis demonstrated that EC patients with lower-level *CCT7* expression had better overall survival (*p* = 0.0081). Gene ontology enrichment indicated that “RNA binding,” “Mitochondrion,” “Translation,” and “Spliceosome” were most significantly enriched potential pathways. Five hub genes, *PSMA5, PSMD14, SNRPB, SNRPG*, and *TXNL4*A, were all significantly upregulated in EC and had a positive correlation with *CCT7*.

**Conclusions:** *CCT7* may be involved in EC development by excessively activating tumor cell function to promote MI or distant/nodal metastasis, which may contribute to the prognosis of EC patients.

## Introduction

Endometrial cancer (EC) is the fourth highest malignant tumor in women and the most common gynecologic cancer of the female reproductive system in the United States, with an overall incidence of 4.4% around the world in 2018 (1, 2). When diagnosed at an early stage, EC is highly curable and has excellent overall 5-year survival rates (3). Although the overall prognosis is better than that of other cancer types, many women (especially young women) have aggressive neoplasms and require a hysterectomy, resulting in a loss of fertility and menstrual function and, accordingly, in physical and mental disability (4).

The International Federation of Gynecology and Obstetrics (FIGO) proposed that EC should be surgically staged, which comprises total hysterectomy, bilateral salpingo-oophorectomy, cytologic washings, and pelvic and para-aortic lymphadenectomy (5). A reliable risk stratification of EC could help to plan a therapeutic schedule and predict the clinical outcomes for EC patients. The risk classification of EC is mainly according to tumor histology, tumor grade, and myometrial infiltration (MI) depth (6, 7). Tumor histology and histological grade may be evaluated preoperatively by endometrial biopsy. The MI depth of EC has a close relationship with lymph node involvement and distant metastasis and is the most important risk factor in apparent early-stage EC, but it is difficult to determine preoperatively (8–10). Therefore, based on comprehensive MI assessment preoperatively, it may assist in better planning of surgical procedures and avoiding unnecessary lymph node dissections (11). Currently, magnetic resonance imaging (MRI) and transvaginal ultrasound (TVS) are the commonest techniques for evaluating preoperatively the depth of MI. However, there are still some controversies and limitations on these techniques in the evaluation of the depth of MI by the EC (12, 13). Thus, it is necessary to develop new methods to assist in comprehensively assessing the depth of MI.

The eukaryotic cytoplasmic chaperonin-containing TCP-1 (CCT), also called TRiC (TCP1 ring complex), is a complex composed of two back-to-back stacked hetero-octameric rings; each ring is constituted by eight different types of subunits (CCTα, β, γ, δ, ϵ, ζ, η, θ; CCT1 to CCT8 in yeast) (14, 15). The eukaryotic chaperonin CCT is involved in the folding of cytoskeletal proteins (actins and tubulins) in an ATP dependent approach (16, 17). In our previous study, we identified that the CCT7 might be closely associated with EC by using isobaric tags for relative and absolute quantitation (iTRAQ)-based proteomic analysis (*p* = 0.02). In the further experiment, our results revealed that the mRNA expression of *CCT7* was significantly higher in EC tissues than normal pericarcinous tissue (*p* < 0.001, *n* = 10) (18). Therefore, in this study, we aimed to detect the CCT7 expression in EC tissues and further explore the developmental mechanism of EC at the cellular level. Bioinformatics methods were also used to insight into potential molecular pathways.

## Materials and Methods

### Tissue Sample Collection

This retrospective study was approved by the Ethics Committees of Xiangya Hospital, Central South University. Patients were fully informed of the study and provided consent before specimen collection. A total of 87 EC specimens from consecutive patients (cancer and adjacent normal tissues) were confirmed by post-operative pathological diagnosis from March 2015 to November 2015 at Xiangya Hospital Central South University. For all patients, relevant clinical data were collected and checked again for confirmation. The age of patients ranged from 31 to 70 years, and mean age was 51.3 ± 12.2 years. A total of 75 cases were endometrioid adenocarcinoma, 5 were adenosquamous carcinoma, 3 were serous papillary adenocarcinoma, 2 were clear cell carcinoma, and 2 were mucinous carcinoma. According to 2009 FIGO guidelines (5) for the surgical staging of EC, 32 were Ia, 36 were Ib, 5 were II, 12 were III, and 2 were IV. Histopathological grading was as follows: 49 cases were G1, 33 cases were G2, and 5 cases were G3.

### Immunohistochemistry (IHC)

Specimens were fixed in 10% formalin, embedded in paraffin, and sectioned. Two experienced pathologists made the histological diagnosis, and CCT7 expression was evaluated using SP Immunohistochemistry Kits (Abcam Ltd., Cambridge, UK). Results were evaluated according to the following criteria (where brown staining of the cytoplasm and cell membrane indicated positive results) based on the degree of positive staining: weakly positive (+), 1 point; positive (+), 2 points; strongly positive (+ + +), 3 points. Additionally, based on the percentage of positive cells, they were scored as follows: <25% positive cells (+), 1 point; 25–50% (+), 2 points; ≧ 50% (+ + +), 3 points; no positive cells indicated a negative result. Finally, a comprehensive indicator was calculated by summing the two scores, where ≦ 3 points was defined as negative, 4–6 points was interpreted as positive, and > 6 points was interpreted as strongly positive.

### Western Blotting Analysis

Proteins were isolated from EC tissues via NP-40 lysis buffer (Abcam Ltd., Cambridge, UK) and then separated in 12% SDS-PAGE gels and blotted on nitrocellulose membranes. The filters were hybridized with polyclonal anti-CCT7 (Abcam Ltd., Cambridge, UK) at 4°C overnight, followed by incubation with the secondary anti-rabbit (Abcam Ltd., Cambridge, UK) for 1 h at room temperature. Anti-Tubulin (Abcam Ltd., Cambridge, UK) was used as the loading control. Gray-scale values were analyzed using the ImageJ software and were also described previously (19).

### Cell Culture and Transfection

Endometrial cancer (Shanghai Zhongqiaoxinzhou Biotech, ZQ0472) and RL95-2 (Shanghai Zhongqiaoxinzhou Biotech, ZQ0362) cell lines were cultured in Dulbecco's Modified Eagle's Medium (Hyclone) supplemented with 5% fetal bovine serum (FBS, Gibco), 300 mmol/L l-glutamine (Hyclone), 5 μg/mL bovine insulin (Hyclone), 10,000 units/mL penicillin (Hyclone), and 10,000 μg/mL streptomycin (Hyclone) at 37°C under 5% CO_2_. The role of *CCT7* in Ishikawa and RL95-2 EC cells was examined using siRNA-mediated *CCT7* knockdown. For this analysis, 50, 100, and 200 μM siRNA targeting *CCT7* (*CCT7*-Homo-914: 5′-CCACACAGUUGAGGAUUAUTT-3′, 5′-AUAAUCCUCAACUGUGUGGTT-3′; *CCT7*-Homo-986: 5′-CCAUCAUUCUGGAGCCAAATT-3′, 5′-UUUGGCUCCAGAAUGAUGGTT-3′; or non-targeting negative control siRNA 5′-UUCUCCGAACGUGUCACGUTT-3′, 5′-ACGUGACACGUUCGGAGAATT-3′; Sangon Bio-technology Co. Ltd., Shanghai, China) and Dharma FECT reagent (Thermo Fisher Scientific, Waltham, MA, USA) were transfected into cells according to the manufacturer's instructions. After 48 h, the expression of *CCT7* was evaluated by qRT-PCR methods described previously (20), and the best *CCT7* siRNA, i.e., the siRNA resulting in the lowest *CCT7* expression level, was selected. Then, Ishikawa and RL95-2 cells were transfected with *CCT7*-targeting siRNA, and cell proliferation, apoptosis, cell cycle, migration, and colony formation assay were examined.

### Cell Proliferation Assay

Cell proliferation was determined using an MTT assay. Briefly, cells (5 × 10^3^) were plated on 96-well plates for 24 h and then cultivated for 24, 48, and 72 h. By metabolic conversion of MTT dye, viable cell densities were determined. Absorbance was read at 490 nm to evaluate assay results.

### Cell Apoptosis Assay

Cell apoptosis was determined using an Annexin V assay as described previously (21). After transfection and/or lidocaine treatment, cells were collected, washed, and suspended in Annexin V-binding buffer. FITC-conjugated Annexin V and propidium iodide (PI; Beyotime, Haimen, China) were added to cells successively. After incubation, Annexin V-binding buffer was added, and cells were analyzed using a FAC Scan Flow Cytometer.

### Cell Cycle Analysis

After transfection and/or lidocaine treatment, cells were harvested after trypsinization. Then, cells were rinsed three times with buffer solution, the concentration was adjusted to 1 × 10^6^ cells/mL, and the Cycle TEST PLUS DNA Reagent Kit (Becton Dickinson, Franklin Lakes, NJ, USA) was used according to the manufacturer's instructions. Cell cycle status was analyzed by flow cytometry using PI. The PI fluorescence intensity of 10,000 cells was measured for each sample.

### Cell Migration Assay

Ishikawa and RL95-2 cells were treated with 0.25% trypsin and suspended in serum-free medium. Ten thousand cells were added to each Transwell and serum-free medium was added to reach 100 μL. The lower chamber was supplemented with 10% fetal bovine serum and 1,640 medium, followed by cultivation for 48 h in an incubator. The broth in each well was discarded, and cells were washed twice with phosphate-buffered saline (PBS). The surfaces of cells were wiped with wet cotton and fixed with acetone: methanol (1:1) at room temperature for 20 min. After cells were washed twice with PBS, they were stained for 15 min with 0.1% crystal violet and washed with PBS three times or more. Finally, images were obtained under an inverted microscope. Absorbance was read at 550 nm to evaluate assay results.

### Cell Colony Formation Assay

As described previously (22), Ishikawa and RL95-2 cells in logarithmic growth phase were treated with 0.25% trypsin and suspended in 10% FBS medium. Then, cells were seeded in a six-well plate with 1 ml of complete medium (500 cells per well) and cultured at 37°C under 5% CO_2_ for 2–3 weeks until the formation of eye-visible cell colony. After washing twice with PBS, cells were fixed with 1 ml 4% paraformaldehyde, and then stained with 0.5% crystal violet for 30 mins. Remove the dye with flow water and dry in air, obtain the image and count the cell colonies.

### Bioinformation Analysis

The *CCT7* expression data of UCEC (Uterine Corpus Endometrial Carcinoma) and normal tissue were carefully downloaded from the TCGA Data Portal website (http://cancergenome.nih.gov). Co-expressed genes of *CCT7* in UCEC were collected from MEM (http://biit.cs.ut.ee/mem), UALCAN (http://ualcan.path.uab.edu), and GEPIA (http://gepia.cancer-pku.cn) for further evaluation. Gathered genes were analyzed using bioinformatics. The enrichment of functions and signaling pathways of the target genes were analyzed in Enrichr (https://amp.pharm.mssm.edu/Enrichr/). The String database (http://www.string-db.org) was applied to construct the protein-protein interaction (PPI) network for the hub gene identification. Moreover, hub genes were selected to obtain their expression and correlation with *CCT7* in UCEC.

### Statistical Analysis

All results are expressed as means ± standard deviation (SD) from three independent experiments. The chi-square test was used to compare positive staining rates between subgroups, and the one-way and two-way ANOVA analysis of variance were used to compare other data implemented in SPSS 18.0. GraphPad Prism was applied to acquire the figure and receiver operating characteristic curves (ROCs). *p* < 0.05 was considered statistically significant.

## Results

### Overexpression of CCT7 in EC Tissues

In our previous study, we found that mRNA expression of *CCT7* significantly higher in EC tissues than in the normal pericarcinous tissue (*p* < 0.001, *n* = 10) (18). To further re-confirm the association of CCT7 expression between EC and the adjacent tissue, we investigated the CCT7 protein expression in 87 EC and 72 adjacent normal endometrium tissues by IHC. Overall, the CCT7-positive expression showed a brown staining of the cytoplasm and cell membrane. The criteria of scoring for IHC results were described in M&M; CCT7-positive cell rates had a significant difference between EC (Figures 1B,C) and adjacent normal endometrium tissues (Figure 1A) (67.8 vs. 51.4%, *p* = 0.035), and for CCT7 strongly positive cell rates, it also had a significant difference (50.7 vs. 33.3%, *p* = 0.033). Correlations between CCT7 expression and clinicopathological features in patients with EC are summarized in Table 1. There was a statistical significance between CCT7 strongly positive expression and the FIGO pathological stage [III/IV (71.4%) vs. I/II (39.7%), *p* = 0.029] of EC. Meanwhile, the CCT7 protein level from 13 EC patients with different FIGO stage was evaluated by WB. We observed a pronounced up-regulation of CCT7 protein in patients with a more advanced FIGO (II-IV) stage compared to those with a lower FIGO stage and normal EC (*p* < 0.0001, Figures 1D,E). Notably, the strongly positive CCT7 expression rates differed significantly between the deep MI group (>1/2) and the superficial MI group (≤1/2) (65.0 vs. 38.8%, *p* = 0.039), and the AUC of the CCT7 expression of EC for FIGO stage and depth of MI was 0.8502 (*p* < 0.0001, Figure 1F) and 0.8694 (*p* < 0.0001, Figure 1G), respectively. Collectively, these results suggested that CCT7 was involved in the process of muscle invasive or distant/nodal metastasis of EC. However, there were no differences between the groups in age, menstrual status, histological grade, and pathological type (Table 1).

**Figure 1:** CCT7 Overexpression in Carcinous Tissue. Immunohistochemistry assay for CCT7 in pericarcinous tissue **(A)** and carcinous tissue (**B**: 20x and **C**: 40x). Western blotting assays were used to evaluate the expression of CCT7 level in the samples from EC patients **(D)**, quantification also performed **(E)**. Receiver operating characteristic curves (ROCs) were used to analyzed the association between CCT7 expression and FIGO stage and MI depth **(F,G)**. ****p < 0.0001, all values represent Mean ± S.D.

**Table 1:** Correlations between CCT7 and clinicopathological features in patients with endometrial cancer.

**Characteristic**	**Cases**	**CCT7**	**CCT7**	***P-*value**
		**+(%)**	**–(%)**	
**Age(years)**				
<60	15	9 (60.0)	6 (40.0)	0.194
≥60	72	30 (41.7)	42 (58.3)	
**Menopause**				
Yes	42	23 (54.8)	19 (45.2)	0.072
No	45	16 (35.6)	29 (64.4)	
**Tissue type**				
Carcinous	87	39 (50.7)	38 (49.3)	0.033^*^
Pericarcinous	72	24 (33.3)	48 (66.7)	
**Pathological stage**				
I–II	73	29 (39.7)	44 (60.3)	0.029^*^
III–IV	14	10 (71.4)	4 (28.6)	
**Histological grade**				
G1	49	19 (38.8)	30 (61.2)	0.182
G2	33	16 (48.5)	17 (51.5)	
G3	5	4 (80.0)	1 (20.0)	
**Depth of invasion**				
<1/2	67	26 (38.8)	41 (61.2)	0.039^*^
≥1/2	20	13 (65.0)	7 (35.0)	
**Pathological type**				
Endometrioid adenocarcinoma	75	34 (45.3)	41 (54.7)	0.813
Other Types^§^	12	5 (41.7)	7 (58.3)	
**Preoperative chemotherapy**				
Yes	31	16 (51.6)	15 (48.4)	0.344
No	56	23 (41.1)	33 (58.9)	

CCT7+: >6 points, strongly positive; CCT7–: ≤6 points, negative and positive;

§ *other types included (cases/CCT7+/CCT7–): Adenosquamous carcinoma (5/1/4), Serous papillary adenocarcinoma (3/1/2), Clear cell carcinoma (2/1/1), and Mucinous carcinoma (2/2/0); Statistical analyses were performed using Chi-square tests*.

* *P < 0.05 was considered statistically significant*.

### Knockdown of *CCT7* Leaded to Loss-of-Function in EC Cellular Level

In order to explore the *CCT7* function in cellular levels, we performed an RNA interference approach to knock down *CCT7* expression in both Ishikawa and RL95-2 cell lines. Two kinds of siRNA targeting *CCT7* (*CCT7*-Homo-914 and *CCT7*-Homo-986) were transfected into cells as described in M&M; the *CCT7* expression levels were unchanged on transient transfection with the negative control siRNA, whereas *CCT7-*specific siRNA significantly reduced mRNA expression levels in the Ishikawa and RL95-2 cell lines (Figures 2A,B). The best *CCT7* siRNA-986 which resulted in the lowest *CCT7* expression level was selected for subsequent experiment. Upon *CCT7* siRNA-986 transfection, Ishikawa and RL95-2 cells exhibited reduced proliferative activity compared with negative control (*p* < 0.0001) (Figures 2C–F).

**Figure 2:** Knockdown of *CCT7* Decreased the Tumor Cells Proliferation Abilities. qPCR was performed to test the mRNA level of *CCT7* after transferring the *CCT7*-siRNA into Ishikawa and RL95-2 cells **(A,B)**. Proliferative abilities of Ishikawa and RL95-2 cells treated with *CCT7* siRNA-986 were determined using an MTT assay after culturing for 24, 48, 72 h **(C–F)**. *p < 0.05, ****p < 0.0001, all values represent Mean ± S.D.

To further verify whether *CCT7-*downregulation influenced EC cell apoptosis and cell cycle, the flow cytometry was used to detect the proportion of cells in different phases. Cell apoptosis was strikingly promoted by *CCT7* siRNA-986 compared with control in both Ishikawa and RL95-2 cells (Figures 3A–C). In addition, the knockdown of *CCT7* reduced the proportion of cells in the S phase and induced G2/M cell cycle arrest significantly (Figures 3D–F), suggesting that *CCT7* played a positive role in the development of EC.

**Figure 3:** Loss of *CCT7* Increased the Tumor Cells Apoptosis and Decreased G2/M Phase of Cells. Cell apoptosis **(A–C)** and cycle **(D–F)** of Ishikawa and RL95-2 cells treated with *CCT7* siRNA-986 were detected by FAC Scan. **p < 0.01, ***p < 0.001, ****p < 0.0001, all values represent Mean ± S.D.

We performed the Transwell experiments as an independent method to prove the anti-invasion effect of *CCT7* suppression in EC cells. As described in M&M, *CCT7*-targeting siRNA-986 contributed to an obvious reduction of the cell migration capacity of both Ishikawa and RL95-2 cells compared with control siRNA-treated cells (*p* < 0.0001, Figures 4A–D), which indicated that *CCT7* was involved in the processes of tumor cell invasion and metastasis. The cell colony formation also revealed that EC cells treated with CCT7-targeting siRNA-986 formed a lower number of colonies than control siRNA-treated cells (Figures 4E–H). Collectively, these loss-of-function studies demonstrated that the *CCT7*-siRNAs could inhibit tumor cell proliferation and invasion abilities compared with the control.

**Figure 4:** Inhibition of *CCT7* Suppressed the Capacity of Tumor Cells Migration and Colony Formation. Migration **(A–D)** and colony formation **(E–H)** of Ishikawa and RL95-2 cells treated with *CCT7* siRNA-986 were examined. **p < 0.01, ***p < 0.001, ****p < 0.0001, all values represent Mean ± S.D.

### Potential Molecular Pathway Prediction by Bioinformatics

In order to explore the potential molecular pathways about *CCT7* in EC, bioinformatics methods were adopted. As shown in Figure 5A, a cohort of 546 UCEC and 35 non-cancerous adjacent endometrium tissues were obtained from the TCGA database. The results demonstrated that the expression of *CCT7* did not significantly differ in UCEC and adjacent endometrium tissues. Notably, the survival analysis showed that the UCEC patients with a lower (*n* = 135) level *CCT7* expression had better overall survival (OS) than the higher (*n* = 408) group (*p* = 0.0081, Figure 5B), which indicated that *CCT7* could be a potential prognostic marker for EC patients. As shown in Venn, 48 genes were obtained from MEM, 105 genes from UALCAN, and 141 co-expression genes from GEPIA, respectively (Figure 6E). Twelve genes, *CCT4, NHP2, C1QBP, CYC1, SAE1, PHB, MDH2, XRCC6, NME1, IMMT, RAN, STOML2*, were intersected in various platforms; then these genes were used to enrich their function and pathways.

**Figure 5:** Data Analysis from TCGA. *CCT7* expression in normal samples (*n* = 35) and UCEC (*n* = 546) were analyzed based on TCGA **(A)**. Survival analysis was performed to test the effect of *CCT7* expression level on UCEC patient survival **(B)**. UCEC, Uterine Corpus Endometrial Carcinoma.

**Figure 6:** GO Enrichment Analysis of *CCT7* in UCEC. Top ten significant enriched pathways of Molecular Function (MF), Biological Process (BP), Cellular Component (CC), and Kyoto Encyclopedia of Genes and Genomes (KEGG) were presented **(A–D)**. Forty eight co-expression genes of *CCT7* obtained from MEM, 105 genes from UALCAN, and 141 genes from GEPIA were summarized in the Venn **(E)**. Protein-protein interaction (PPI) network was displayed **(F)**.

The gene ontology (GO) enrichment analysis comprised three categories: the molecular function (MF), the biological process (BP) and the cellular component (CC). GO enrichment indicated that *CCT7* was enriched in 80 MF, 153 BP, 59 CC. The 10 most valuable pathways of each category are presented in Figures 6A–C. Among enriched pathways, the most significant pathway was “RNA binding” in MF, “Mitochondrion” in CC and “Translation” in BP. Based on the Kyoto Encyclopedia of Genes and Genomes (KEGG) pathways, the 10 most significant pathways are shown in Figure 6D, of which “Spliceosome” was the most significantly enriched pathway.

The PPI network was displayed (Figure 6F); 10 pairs of hub genes with the highest combined scores were collected from the PPI network (Table 2). Compared with non-cancerous endometrium tissues, the hub genes *PSMA5, PSMD14, SNRPB, SNRPG*, and *TXNL4A* were significantly upregulated in UCEC (*p* < 0.05, Figures 7A–E). Moreover, correlations between hub genes and *CCT7* were analyzed, and all genes were positively correlated with *CCT7* in UCEC (*p* < 0.0001, Figures 7F–J).

**Table 2:** Top 10 pairs of hub genes from the PPI network.

**Node-1**	**Node-2**	**Homology**	**Co-expression**	**Experimentally determined interaction**	**Database annotated**	**Automated text mining**	**Combined score**
SNRPG	SNRPD3	0	0.986	0.993	0.9	0.901	0.999
RRP9	FBL	0	0.804	0.827	0.9	0.832	0.999
SNRPB	SNRPG	0	0.45	0.991	0.9	0.853	0.999
PDCD11	RRP9	0	0.864	0.733	0.9	0.757	0.999
TXNL4A	SNRNP40	0	0.107	0.989	0.9	0.293	0.999
NOP14	RRP9	0	0.879	0.796	0.9	0.755	0.999
SNRPB	SNRPD3	0	0.555	0.992	0.9	0.857	0.999
SNRPG	SNRPC	0	0.634	0.981	0.9	0.624	0.999
PSMD14	PSMA5	0	0.912	0.992	0.9	0.563	0.999
SNRPC	SNRPD3	0	0.868	0.96	0.9	0.842	0.999

**Figure 7:** Hub Genes Identification and the Correlation with *CCT7* in UCEC. The expression of hub genes in UCEC and non-cancerous were analyzed **(A–E)** and their correlation with *CCT7* were also examined **(F–J)**. *p < 0.05, all values represent Mean ± S.D.

## Discussion

EC is one of the most frequent gynecological cancers worldwide (1). The incidence and mortality of EC are rising throughout the developed world with a tendency for onset at a younger age, and this trend is expected to continue mainly due to the increasing prevalence of obesity, hypertension, diabetes, and prolonged life expectancy (23). For purposes of improving treatment and follow-up of EC patients, the importance of various prognostic factors had been extensively studied over the past few decades, including pathological stage, histological type and grade, age, tumor size, and lymphovascular space involvement (5, 24–26). In addition, some tumor biomarkers also had been studied for their potential clinical value in patients with EC, including HE4, chaperonin 10, CA125, CA15.3, CA19.9, CA72.4, CEA, OVX1, and M-CSF (23, 27). However, no good marker was routinely recommended for patients with EC. A study with a large sample is probably needed to validate the independent connection of the abovementioned variables and biomarkers with prognosis.

EC typically spreads by the invasion of the myometrium into the cervix, or via the fallopian tubes to the ovaries or trans-serosal spread to the bladder or bowel (28). The role of preoperative staging is aiming to establish a recurrence risk group to inform surgical management decisions, mainly based on tumor histology, tumor grade, MI depth, and lymph node metastasis (29). The tumor histology and grade may be evaluated preoperatively by endometrial biopsy, but it is difficult to determine the extent of MI accurately using the techniques in clinical practices. MI by the EC was associated with lymph node involvement, and prognostic significance of both for EC patients were well-documented (8, 10). Thus, methods to assess the extent of MI are important. Clinically, TVS is excellent in determining the endometrial thickens, but it is limited in the evaluation of the depth of MI by the EC (13). MRI is considered the most accurate imaging technique for the preoperative assessment of EC due to its excellent soft tissue contrast resolution. However, there are some limitations including the uterine anatomy distorted by leiomyomas, presence of adenomyosis, and the tumor involving a cornu of the uterus (12). Recent meta-analyses (30) had shown that estimated sensitivity and specificity for diagnosing deep MI were 75% [95% confidence interval [CI] = 67–82%] and 82% (95% CI = 75–93%) for TVS, and 83% (95% CI = 76–89%), and 82% (95% CI = 72–89%) for MRI, respectively. However, all studies included in this systematic review were both on high- and low-risk patients for deep MI, which may affect the clinical applicability of both techniques. Therefore, it is necessary to develop new methods to assist in evaluating the extent of MI for a precise determination of prognosis and an accurate tailoring of adjuvant therapy.

To date, there are no molecular markers that could help to assess the depth of MI by the EC. *CCT7*, also known as the *TCP1* ring complex, consists of two identical stacked rings and folds various proteins, and is involved in the folding of cytoskeletal proteins in an ATP dependent approach (16, 31, 32). Based on our results, *CCT7* may have a critical role in the processes of muscle invasion and distant/nodal metastasis in EC development. Our previous proteomics experiments had shown that the *CCT7* gene was differentially expressed between EC and adjacent normal tissues (18), which was re-verified in the present study (*p* = 0.033). Of note, we found that the rate of CCT7 strongly positive cells differed significantly between the two groups, i.e., patients with and without deep MI (*p* = 0.039), along with the ROC (AUC = 0.8502, *p* < 0.0001) between CCT7 expression and MI depth, suggesting that CCT7 was related to MI and it could be a valuable biomarker to evaluate the extent of MI by the EC. Better prognosis of EC patients related to lower pathological stages had been suggested (5). Additional analyses confirmed that CCT7 expression also had an obvious correlation with the pathological stage of patients, as advanced stage (III/IV) EC patients had higher CCT7 strongly positive cell rates and CCT7 protein level compared to lower-stage (I/II) patients (*p* = 0.029 and Figure 1E), same as the ROC (AUC = 0.8694, *p* < 0.0001) between CCT7 expression and FIGO stage, which demonstrated that patients with higher CCT7 expression would have an unfavorable prognosis. Notably, corresponding with the survival analysis based on TCGA data, which showed that the EC patients with lower level *CCT7* expression had better OS (*p* = 0.0081), and *CCT7* had a potential prognostic value for EC patients.

Subsequently, we attempted to validate the potential function and predict the potential molecular pathways of *CCT7* in EC development; the siRNA method to knock down *CCT7* expression in Ishikawa and RL95-2 cell lines was performed. We found diminished proliferation activity, invasion abilities, and colony capacity in both Ishikawa and RL95-2 cells after *CCT7* knockdown. At the same time, further studies revealed that loss of *CCT7* significantly stimulated the cell apoptosis and induced G2/M cell cycle arrest in EC cells. Collectively, *CCT7* expression was considerably correlated to EC cell function, which could affect multiple aspects of tumor cell development. For the bioinformatic analysis, based on TCGA, there was no significance in CCT7 expression between UCEC and normal samples, but the imbalance between the tumor and normal data may cause inefficiency for analysis. In addition, GO enrichment indicated that “RNA binding,” “Mitochondrion,” “Translation,” and “Spliceosome” were most significantly enriched potential pathways. In addition, five hub genes were analyzed from the PPI network, *PSMA5, PSMD14, SNRPB, SNRPG*, and *TXNL4*A, which were all significantly upregulated in UCEC compared to adjacent healthy controls. *PSMA5* and *PSMD14* are the core components of the proteasome complex that participates in numerous cellular processes, including cell cycle progression, apoptosis, or DNA damage repair (33, 34). It was reported that *PSMA5* and *PSMD14* could promote the tumorigenic process and tumor metastasis in various cancers (35, 36). *SNRPB, SNRPG*, and *TXNL4A* are the core components of spliceosome and play a major role in regulating alternative splicing of the pre-mRNA (37, 38). *SNRPB* was reported to promote the non-small cell lung cancer tumorigenesis (39). These five genes were positively correlated with *CCT7* in UCEC, which revealed that *CCT7* may have a similar potential tumorigenic function.

In our present work, we first provided a new method based on CCT7 to assess the extent of MI by EC, and CCT7 could also be a potential biomarker to predict prognosis. However, there are some limitations we have to acknowledge. Firstly, in this retrospective study, we only investigated the CCT7 expression in EC and adjacent normal endometrium tissues, but healthy patients were not included, which may affect the clinical utility of this biomarker. Secondly, although the survival data based on TCGA showed that CCT7 high expression was related to unfavorable outcome in EC patients, due to the lack of direct survival data about CCT7 expression in 87 EC patients included in our study, definitely the predictive value of CCT7 expression in prognosis could not be assessed and further survival analysis was needed. Thirdly, the potential molecular pathway was predicted but further confirmed experiments were needed.

## Conclusion

Collectively, our results provided a new view of the molecular changes in EC. CCT7 may be involved in EC development by excessively activating tumor cell function, invasive ability in particular, to promote MI or distant/nodal metastasis, which may contribute to the prognosis of EC patients.

## Data Availability Statement

Publicly available datasets were analyzed in this study, these can be found in The Cancer Genome Atlas (https://portal.gdc.cancer.gov/).

## Ethics Statement

The studies involving human participants were reviewed and approved by Ethics Committees of Xiangya Hospital, Central South University. The patients/participants provided their written informed consent to participate in this study.

## Author Contributions

NS was responsible for conception, design, quality control of this study, and reviewed and edited the manuscript. LW and WZ performed the experiments, data extraction, statistical analyses, and were major contributors in writing the manuscript. HL and HY participated in experiments and statistical analyses. All authors have read and approved the final version of the manuscript.

## Conflict of Interest

The authors declare that the research was conducted in the absence of any commercial or financial relationships that could be construed as a potential conflict of interest.
